RETRACTED

# An Epidemiological Study of Risk Factors of Thyroid Nodule and Goiter in Chinese Women

**DOI:** 10.3390/ijerph120911608

**Published:** 2015-09-16

**Authors:** Lei Zheng, Wenhua Yan, Yue Kong, Ping Liang, Yiming Mu

**Affiliations:** 1 Department of Endocrinology, Chinese People’s Liberation Army (PLA)General Hospital, 28 Fu Xing Road, Beijing 100853, China; E-Mails: zhenglei79541@163.com (L.Z.); yanwenhua301@163.com (W.Y.); 2 Department of Endocrinology, First Affiliated Hospital of Chinese People’s Liberation Army General Hospital, 51 Fucheng Road, Beijing 100048, China; 3 Department of Interventional Ultrasound, Chinese People’s Liberation Army General Hospital, 28 Fu Xing Road, Beijing 100853, China; E-Mail: kongyue79541@163.com (Y.K.); liangping301@hotmail.com (P.L.); 4 Department of Ultrasound, Beijing Shijitan Hospital, The 9th Clinical Medical College of Peking University, 10 Tieyi Road, Yangfangdian, Haidian District, Beijing 100038, China

**Keywords:** epidemiology, prevalence, risk factor, metabolic syndrome

## Abstract

Thyroid nodule (TN) and goiter are two common disorders of the thyroid. Despite their benign nature, both conditions can be associated with multiple pathologic conditions including thyroid cancer. In this study, we conducted a large-scale epidemiological study in Chinese women to identify the risk factors implicated in the occurrence of TN and goiter. We analyzed demographic data, lifestyle, medical history, body height, weight, waist circumference, body mass index (BMI), blood pressure, serum glucose and lipids. In addition, thyroid ultrasonography was performed for all subjects. Our results showed that age, menopause, waist circumference, BMI, hypertension, dyslipidemia, and hyperglycemia were associated with both TN and goiter. Furthermore, we found that the prevalence of TN was significantly affected by the medical management of hypertension. Our study suggests that postmenopausal Chinese women with advanced age, obesity, diabetes, and hypertension have an increased awareness of thyroid examination in the annual physical check. Conversely, patients with TN and goiter of the same population may have a higher incidence of age- and obesity-related metabolic disorders.

## 1. Introduction

Thyroid nodule (TN) and goiter are two common thyroid disorders that have global influence [1,2,3,4,5]. The presentation of these two conditions range from mild changes in the thyroid structure without clinical manifestations to severe symptoms such as breathing and/or swallowing difficulties that affect life quality and expectancy. In one study, Allan Carlé *et al.* [4] reported approximately 10% of the world population was affected by goiter [4]. Research on the prevalence of TN otherwise reported that it approached 50% when the nodules were detected by ultrasound and/or other radiologic methods [6]. In addition, although TN and goiter have no clinical manifestations in majority of patients, both conditions can be associated with varied pathologic conditions of the thyroid including thyroiditis, endocrine dysregulation, and autoimmune disease [1,2,3]. Furthermore, approximately 18% of toxic nodular goiters are proven cancerous following extensive medical workup [1].

RETRACTED

TN and goiter have multiple known risk factors, which include demographic parameters and clinical history. Age and sex, respectively, correlates with the occurrence, increasing the prevalence of TN and goiter in residents of the United States [7,8].Similar observations were made by the studies conducted in the Chinese populations [9,10]. Interestingly, both diseases have a pattern of female predominance [11,12,13]. The Framingham study conducted on 5217 participants showed that 6.4% of women and 1.5% of men were affected by TN [14]. Another independent research also reported that the highest prevalence of goiter occurred in pre-menopausal females and that the ratio of female/male was greater than 4:1 [15]. Similarly, a Chinese community-based population study revealed that the prevalence of TN in 9533 Chinese adults aged over 40 years is 50.3% in women (odds ratio = 1.951) compared with 39.7% in men [16]. In lifestyle, smoking was identified by multiple studies as predisposing the study population to TN and goiter [17,18]. Furthermore, thyroid volume, a mathematical quantitation of the goiter, was positively correlated with increased body mass index (BMI) [19], and hyperglycemia in patients with impaired glucose metabolism [20]. Finally, incidence of TN and goiter increased in individuals with clinically diagnosed hypertension [16] and diabetes [13].

In this paper, we conducted a large-scale epidemiological study to explore the risk factors of TN and goiter in Chinese women.

## 2. Materials and Methods

### 2.1. Subjects

The study was conducted in Daxing district of Beijing, China from August to December in 2013. The study was part of a larger ongoing longitudinal study designed to investigate the prevalence of TN in community-based populations in China. A total of 6323 volunteers received the questionnaire and were examined by thyroid ultrasonography (US). All participants were 18 years or older. Pregnant women and those with severe cardiac, hepatic, or renal disease and so on were excluded. Participants with one or more of the following characteristics were also excluded from the study: (1) history of thyroid procedures such as thyroid surgery or radiotherapy in thyroid, head or neck; ongoing medical treatments including thyroxine, iodine, amiodarone, or anti-thyroid medications (*n* = 181); (2) subjects with incomplete data in questionnaire, or with incomplete physical examination and/or laboratory tests; participants with data acquisition errors (*n* = 795); and (3) males (*n* = 2263). Finally, 3084 females were analyzed by the study. All participants provided informed consent to the study initiative by the residential committees.

RETRACTED

### 2.2. Anthropometric Measurements

Each participant completed a detailed questionnaire for demographic data, lifestyle, and medical history. Demographic data included gender, age, education, and marital status. Education was classified into six categories: uneducated, elementary, middle school, high school, junior college, and undergraduate and above. Marital status included married, and divorced or widowed. Lifestyle included salt intake, smoking, alcohol consumption, seafood intake, and exercise. Salt intake was classified into three categories: mild, medium, or high. Smoking history included three categories: never, prior, or active, with the latter referring to at least one cigarette per day for the last six months. Alcohol consumption was also classified into three categories: never, prior, or active, with active consuming alcohol at least once a week for the last six months. Dietary intake of seafood included never, occasional, or frequent (defined as no less than three times per week). Exercise intensity in the last six months was defined according to the following criteria: mild, physical activities of 10 min that did not result in sweating, tachycardia, or tachypnea; medium, physical activities of 10 min resulting in light sweating and/or mild tachycardia and tachypnea; and high, physical activities of 10 min resulting in profuse sweating and/or severe tachycardia and tachypnea. Medical history included hypertension, dyslipidemia, diabetes mellitus, menstrual status, and thyroid diseases. Participants were measured for body height, weight, waist circumference, and BMI (kg/m^2^). Blood pressure was measured three times with an automated blood pressure monitor (HEM-7117 OMRON Co. Inc, Dalian, China) on the right upper arm after the participants had rested for minimal 5 min. Average value of the triple readings was used for the study.

### 2.3. Laboratory Medicine Measurement

All participants were fasted overnight. Venous blood was collected and tested. Oral glucose tolerance test (OGTT) with 75 g of glucose was performed for participants without diagnosed diabetes or receiving hypoglycemic medications. Fasting plasma glucose (FPG), 2 h postprandial glucose (PPG), total cholesterol (TC), triglyceride (TG), high-density lipoprotein cholesterol (HDL-C), and low-density lipoprotein cholesterol (LDL-C) were analyzed by a HITACHI automated biochemical analyzer (7600 HITACHI Ltd, Tokyo, Japan).

RETRACTED

### 2.4. Thyroid Ultrasound

Thyroid ultrasound examination was performed using a portable SonoScape ultrasound device with 5–12 MHz linear probe, or a GE LOGIQ e device with 4–10 MHz linear probe. Volume of each thyroid lobe was determined by the Ellipsoid formula: Volume (mL) = Length (cm) × Width (cm) × Thickness (cm) × 1/6 Л. Goiter is defined as the total volume larger than 18 mL in women and 25 mL in men [21]. Double blinding was applied to the test subjects and ultrasound technologists to avoid biases in the interpretation of results.

### 2.5. Definitions and Normal Values

Hypertension was defined according to the European Society of Hypertension (ESH) 2013 guidelines as systolic blood pressure (SBP) ≥ 140 mmHg and/or diastolic blood pressure (DBP) ≥ 90 mmHg. Hypertensive patients were defined as participants meeting the above criteria or taking oral anti-hypertensive medications. Hyperglycemia was classified into pre-diabetes and diabetes according to the American Diabetes Association 2013 guidelines. Pre-diabetes has high risk in developing diabetes and complications. It was diagnosed by any of the following criteria: impaired fasting glucose (IFG): FPG 5.6–6.9 mmol/L; impaired glucose tolerance (IGT): 2 h PPG in 75 g OGTT 7.8–11.0 mmol/L. Diabetes was diagnosed by FPG ≥ 7.0 mmol/L or 2 h PPG in 75 g OGTT ≥ 11.1 mmol/L. Diabetic patients were defined as participants meeting the above criteria or taking hypoglycemic medications. Dyslipidemia was defined by the International Diabetes Federation (IDF) as TG level ≥ 150 mg/dL (1.7 mmol/L) or patients receiving medical management for lipid abnormalities; and HDL-C < 40 mg/dL (1.03 mmol/L) in males and < 50mg/dL (1.29 mmol/L) in females or patients receiving medical management. According to the International Diabetes Federation (IDF) 2005 guidelines, waist circumference ≥ 90 cm for men and ≥ 80 cm for women in the Chinese population indicate obesity. According to WHO, overweight is defined as BMI ≥ 25 kg/m^2^, whereas obesity is defined as BMI ≥ 30 kg/m^2^. Hyperuricemia was diagnosed when the serum uric acid exceeded 7.0 mg/dL.

### 2.6. Statistics Analysis

Categorical variables were analyzed using chi-square test or fisher’s exact test. Numeric variables were compared using t test if in normal distribution and Wilcoxon Rank-Sum test if not in normal distribution. Potential risk factors of TN and goiter were analyzed by logistic multiple stepwise regression with P-value at 0.1 of entry and remove variables. The variables in our study included age, parity, alcohol consumption, smoking, education, seafood intake, salt intake, hypertension, diabetes, menopause, dyslipidemia, and BMI. In all tests, *p* value < 0.05 was deemed statistically significant.

RETRACTED

## 3. Results

### 3.1. Demographic Data, Lifestyle, and Medical Characteristics of the Study Population

Based on the criteria of inclusion and exclusion, total 3084 (out of 6323 participants) subjects were analyzed by the study (Table 1). Demographic data included age, education, and marital status. Within the study population, participants less than 30 years of age were 3%, near 40 were 11%, near 50 were 25%, near 60 were 33%, near 70 were 24%, and older than 70 were 5%. The age showed a normal distribution with the median age being 52. With regard to education, 7% participants received no formal education, 22% graduated from elementary school, 43% graduated from middle school, 21% graduated from high school, 5% graduated from junior college, and 2% completed undergraduate studies or above. Nearly 100% of the study population was currently married. The lifestyle included drinking, smoking, seafood intake, exercise, and salt intake. Of the study population, 96% denied drinking, 1% admitted prior drinking, and 3% was actively drinking. Compatible with this data, 94% participants denied smoking, 1% had prior smoking history, and 5% was smoking at present. In seafood consumption, 15% of the study population reported rarely, 79% occasionally, and 6% frequently had seafood in their diet. Exercise was classified into high, modest, or low intensity, for which the study population responded with 1%, 8% and 92%, respectively. Lastly, with reference to salt intake, 23% of the study group had low, 47% had medium, and 30% had high salt in their diet. Medical characteristics included parity, menopause, BMI, waist circumference, hypertension, hyperglycemia, dyslipidemia, and hyperuricemia. Forty-six percent of the women had one child, 50% had two to three, and 4% had no less than four children. Forty present of the study subjects were actively menstruating, and 60% had reached their menopause. As stated earlier, overweight/obesity was defined as BMI ≥ 25 kg/m^2^. In the study group, 32% participants were normal, and 68% were overweight/obese. This was consistent with another obesity parameter, the waist circumference. Of the female participants, 21% showed less than (normal) and 79% showed no less than 80 cm (obese) in length.

### 3.2. Clinical and Demographic Features of TN and Goiter

We next examined various clinical and demographical features of TN and goiter (Table 1 and Table 2). For TN, we observed a significant relationship (*p* < 0.05) with the following variables: education level, age, and parity, menopause, smoking, high salt intake, seafood consumption, BMI, waist circumference, hypertension, hyperglycemia, and dyslipidemia. The prevalence of TN increased with the parity, while declined with the educational level. We found no association with marital status, drinking, exercise, and hyperuricemia. For goiter, we observed a significant association (*p* < 0.05) with menopause, waist circumference, BMI, hypertension, dyslipidemia, and hyperglycemia. Interestingly, age of the population displayed a discordant association with goiter. At, before, or near 60 years of age, it showed a positive relationship, and after 60 a negative relationship. Other factors not relevant to goiter included education level, marital status, parity, drinking, smoking, seafood intake, salt intake, exercise and hyperuricemia. Taken together, the factors associated with both TN and goiters were menopause, waist circumference, BMI, hypertension, dyslipidemia, and hyperglycemia.

RETRACTED

**Table 1:** Characteristics of the study population and TN.

Variables	TN		Variables	TN	
	TN/Total Subjects (%)	*p* Value		TN/Total Subjects (%)	*p* Value
Education		<0.001	Age (%)		<0.001
uneducated	145/219 (66.2)		<30	23/81 (28.4)	
elementary	407/682 (59.7)		~40	117/ 333 (35.1)	
middle school	660/1317 (50.1)		~50	337/758 (44.5)	
high school	321/642 (50.0)		~60	571/1026 (55.7)	
junior college	67/160 (41.9)		~70	467/739 (63.2)	
undergraduate and above	18/64 (28.1)		≥70	103/147 (70.1)	
Marital status (%)		0.336	BMI		<0.001
married	1609/3069 (52.4)		<25	465/975 (47.7)	
divorced or widowed	9/15 (60)		≥25	1153/2109 (54.7)	
Parity		<0.001	Seafood consumption		0.002
1	644/1420 (45.4)		never	264/448 (58.9)	
2 or 3	897/1550 (57.8)		occasional	1259/2420 (52.0)	
≥4	75/112 (67.0)		frequent	88/198 (44.4)	
Menopause (%)		<0.001	Hypertension (%)		<0.001
no	514/1236 (41.6)		no	765/1671 (45.8)	
yes	1104/ 1848 (59.7)		yes	853/1413 (60.4)	
Alcohol consumption		0.396	Smoking history		0.002
never	1557/2969 (52.4)		never	1496/2897 (51.6)	
prior	11/16 (68.8)		prior	28/43 (65.12)	
active	50/99 (50.5)		active	94/144 (65.28)	
Waist circumference		<0.001	Dyslipidemia (%)		0.009
<80	253/637 (39.7)		no	772/1541 (50.1)	
≥80	1365/2447 (55.8)		yes	846/1543 (54.8)	
Hyperglycemia level		<0.001	Salt intake		0.027
normal	649/1351 (48.0)		mild	355/707 (50.2)	
pre-diabetes	520/1024 (50.8)		medium	738/1438 (51.3)	
diabetes	449/709 (63.3)		high	521/928 (56.1)	
Exercise intensity		0.361	Hyperuricemia (%)		0.102
high	7/19 (36.8)		no	1534/2942 (52.1)	
medium	118/225 (52.4)		yes	84/142 (59.2)	
mild	1424/2680 (53.1)				

RETRACTED

**Table 2:** Characteristics of the Study Population and Goiter.

Variables	Goiter		Variables	Goiter	
	Goiter/Total Subjects (%)	*p* Value		Goiter/Total Subjects (%)	*p* Value
Education		0.077	Age (%)		<0.001
uneducated	23/219 (10.5)		<30	2/81 (2.5)	
elementary	67/682 (9.8)		~40	12/333 (3.6)	
middle school	117/1317 (8.9)		~50	60/758 (7.9)	
high school	54/642 (8.4)		~60	118/1026 (11.5)	
junior collage	7/160 (4.4)		~70	66/739 (8.9)	
undergraduate and above	1/64 (1.6)		≥70	11/147 (7.5)	
Marital status (%)		0.837	BMI		<0.001
married	267/3069 (8.7)		<25	36/975 (3.7)	
divorced or widowed	2/15 (13.3)		≥25	233/2109 (11.1)	
Parity		0.184	Seafood consumption		0.204
1	110/1420 (7.8)		never	44/448 (9.8)	
2 or 3	147/1550 (9.5)		occasional	212/2420 (8.8)	
≥4	12/112 (10.7)		frequent	11/198 (5.6)	
Menopause (%)		0.01	Hypertension (%)		<0.001
no	88/1236 (7.1)		no	114/1671 (6.8)	
yes	181/1848 (9.8)		yes	155/1413 (11.0)	
Alcohol consumption		0.307	Smoking history		0.314
never	259/2969 (8.7)		never	247/2897 (8.5)	
prior	3/16 (18.8)		prior	5/43 (11.6)	
active	7/99 (7.1)		active	17/144 (11.8)	
Waist circumference		<0.001	Dyslipidemia (%)		0.004
<80	23/637 (3.6)		no	112/1541 (7.3)	
≥80	246/2447 (10.1)		yes	157/1543 (10.2)	
Hyperglycemia level		0.001	Salt intake		0.194
normal	93/1351 (6.9)		mild	50/707 (7.1)	
pre-diabetes	93/1024 (9.1)		medium	135/1438 (9.4)	
diabetes	83/709 (11.7)		high	83/928 (8.9)	
Exercise intensity		0.299	Hyperuricemia (%)		0.426
high	0/19 (0.0)		no	254/2942 (8.6)	
medium	17/225 (7.6)		yes	15/142 (10.6)	
mild	242/2680 (9.0)				

### 3.3. Obesity and Dyslipidemia Are Associated with Increased Prevalence of TN and Goiter

From the above analyses, we concluded that menopause, waist circumference, BMI, hypertension, dyslipidemia, and hyperglycemia were significantly related to TN and goiter. To further determine the relationship, we directly compared the participants with or without TN or goiter, and their waist–hip ratio (WHR), BMI, TC, TG, and menopausal age. Note that other metabolic parameters such as HDL and FPG were excluded from the analysis given that they showed large variations in our study. Shown in Table 3, WHR, BMI, and TG had a statistically significant association (*p* < 0.01) with both TN and goiter, and TC only associated (*p* < 0.001) with TN. Note that with this method, we did not observe statistical significance for median menopausal age (approximately 49 years of age).

**Table 3:** Relationship between WHR, BMI, TC, TG and Menopause with TN or Goiter.

Parameters	TN			Goiter			
	TN	Non-TN	*p* Value		Goiter	Non-Goiter	*p* Value
WHR	0.88 ± 0.07	0.86 ± 0.09	0.000		0.88 ± 0.06	0.87 ± 0.08	0.000
BMI (kg/m^2^)	27.45 ± 4.05	26.83 ± 4.50	0.000		29.04 ± 3.84	26.98 ± 4.11	0.000
TC (mmol/L)	5.30 ± 1.62	5.09 ± 1.07	0.000		5.25 ± 1.04	5.20 ± 1.42	0.290
TG (mmol/L)	1.6 ± 1.13	1.52 ± 1.25	0.000		1.76 ± 1.53	1.55 ± 1.15	0.002
Menopause (age)	49.55 ± 3.88	49.30 ± 4.33	0.170		49.19 ± 4.10	49.47 ± 4.07	0.532

RETRACTED

### 3.4. The Relationship of Medical Management of Comorbidities with TN and Goiter

Next, we examined whether medical management of aforementioned comorbidities and risk factors could be associated with the prevalence of TN and goiter. We observed in our TN study group statistical significance (*p* < 0.05) of anti-hypertensive therapy. Medical therapies in patients with diabetes and dyslipidemia, and estrogen supplementation in postmenopausal participants, however, had no statistically significant impact on either TN or goiter (Table 4).

**Table 4:** Relationship of Medical Management of Comorbidities with TN or Goiter.

Variables	TN		Goiter	
	TN/Total Subjects (%)	*p* Value	Goiter/Total Subjects (%)	*p* Value
Hypertension (%)		0.015		0.157
treated	572/912 (62.7)		108/912 (11.8)	
untreated	281/501 (56.1)		47/501 (9.4)	
Diabetes (%)		0.649		0.593
treated	210/327 (64.2)		36/327 (11.0)	
untreated	239/382 (62.6)		47/382 (12.3)	
Dyslipidemia (%)		0.099		0.5664
treated	101/166 (60.8)		19/166 (11.5)	
untreated	745/1377 (54.1)		138/1377 (10.0)	
Menopause (%)		0.566		0.679
treated	4/9 (44.4)		0/9 (0.0)	
untreated	1039/1748 (59.4)		169/1748 (9.7)	

### 3.5. Stratification of Associations and Comorbidities in TN and Goiter

Finally, we stratified the associations and identified significant comorbidities from our studies. Age directly associated with TN and goiter with statistical significance (*p* < 0.001 and *p* < 0.01, respectively). The risk of TN was increased by 3% with an age increased by every one year, by 18% with an age increased by every five years, and by 39% with an age increased by every 10 years (Table 5). Likewise, age over 40 was a strong predictor of goiter (odds ratio (OR) of age 40–50, 50–60, ≥60 *vs.* <40 was 1.871 (95% CI: 1.023–3.423), 2.531 (95% CI: 1.409–4.544), and 1.706 (95% CI: 0.925–3.148), respectively). Additionally, women with diabetes and hypertension had 1.328 (95% CI: 1.105–1.597) and 1.277 (95% CI: 1.087–1.500) times the risk of developing TN. BMI also strongly predicted the likelihood of developing goiter (OR = 2.859, 95% CI: 1.972–4.145).

**Table 5:** Analysis of associations for TN or Goiter.

Variables	TN		Variables	Goiter	
	OR (95% CI)	*p* Value		OR (95% CI)	*p* Value
Age		0.000	Age		0.003
unit = 1	1.034 (1.026, 1.042)		40–50 *vs.*<40	1.871 (1.023, 3.423)	
unit = 5	1.183 (1.139, 1.229)		50–60 *vs.* <40	2.531 (1.409, 4.544)	
unit = 10	1.399 (1.297, 1.509)		≥60 *vs.* <40	1.706 (0.925, 3.148)	
Diabetes		0.003	BMI		0.000
yes *vs.* no	1.328 (1.105, 1.597)		≥25 *vs.* <25	2.859 (1.972, 4.145)	
Hypertension (Yes *vs.* No)		0.003	Hypertension		0.065
yes *vs.* no	1.277 (1.087, 1.500)		yes *vs.*no	1.29 (0.984, 1.705)	
Salt intake		0.098			
medium *vs.* mild	1.159 (0.962, 1.396)				
high *vs.* mild	1.247 (1.018, 1.526)				

RETRACTED

## 4. Discussion

TN and goiter are frequent screening findings wherein patients may or may not present with clinical symptoms and/or abnormal laboratory tests.

In this study, we conducted a large-scale observational study in the Chinese female population, aimed to further identify the risk factors of its occurrence. Our data suggest that menopause, waist circumference, BMI, hypertension, dyslipidemia, and hyperglycemia are associated risk factors. Our findings investigated these similar factors with earlier studies performed in other populations [16,22,23,24]. It is worth noting that most identified risk factors are components of the metabolic syndrome, a disorder of energy utilization and storage manifested as conditions such as hyperglycemia, dyslipidemia, arterial hypertension, and obesity. Metabolic syndrome is a major health issue in Western countries, with data estimating the prevalence in the United States to be 34% [25]. With the economic development and changes in life habits in recent years, it has become a growing concern in the Chinese population [26]. Recent surveys show that metabolic syndrome occurs in 12.7% of Chinese males and 14.2% of Chinese females, and the incidence of cardiovascular disease was high in an epidemiologic study in 11 provinces in China [27]. It was long speculated that components of the metabolic syndrome might contribute to thyroid conditions including TN and goiter, yet the definitive conclusion could not be drawn due to the insufficiency of data. In one report, abdominal obesity was associated with thyroid disease [28]. In another study, prevalence of dyslipidemia increased accordingly to higher thyroid-stimulating hormone (TSH) concentrations [29]. In contrast to studying one single metabolic disorder, our study included most components of the metabolic syndrome, thereby providing the one-step-further evidence in the strong association with the two thyroid disorders.

TN is more frequent in females than in males [14]. This has promoted us to choose Chinese women as the study population. In our study, we observed an association between menopause and TN. We excluded estrogen and estrogen use based on the fact that few postmenopausal Chinese women take estrogen containing medications, even though the literature from another country indicated that estrogen contributed to the occurrence of TN [22]. Concerning age, our speculation is that advanced age contributes to the high rate of TN in postmenopausal females.

RETRACTED

Nonetheless, there are other implicated factors that are worth further investigation. For instance, smoking was known to precipitate metabolic syndrome [30] and some thyroid pathological conditions [31]. Our female study group was less engaged in smoking compared to the males of the same geographic area. Furthermore, Hyperuricemia is a known etiologic factor of gout. It has recently been recognized for its involvement in metabolic syndrome [32,33]. In our survey, however, we did not identify a strong association with TN and goiter. Future work is needed to determine whether the characteristics of this study population were involved in generating this observational disagreement. Furthermore, our study was conducted during work hours on workdays when the younger populations were at work or study; the recruited participants thus largely represent the older populations (as reflected by a median age of 52). It is possible that some of the findings may not be applicable to the general community-based population in China.

## 5. Conclusions

Together, our study is one of the first large-scale epidemiological studies of risk factors in the occurrence of TN and goiter in Chinese women. We propose that postmenopausal patients in the Chinese population with advanced age and obesity have an increased awareness of weight reduction and control of metabolic symptoms, and should be examined for TN and goiter during their annual physical examination. Conversely, patients of the same population with confirmed TN and goiter may have a higher incidence of age- and obesity-related disorders such as hypertension and diabetes.

## References

[1] Smith J.J., Chen X., Schneider D.F., Nookala R., Broome J.T., Sippel R.S., Chen H., Solorzano C.C. (2013). Toxic nodular goiter and cancer: A compelling case for thyroidectomy. Ann. Surg. Oncol..

[2] Reverter J.L., Fajardo C., Resmini E., Salinas I., Mora M., Llatjós M., Sesmilo G., Rius F., Halperin I., Webb S.M. (2014). Benign and malignant nodular thyroid disease in acromegaly. Is a routine thyroid ultrasound evaluation advisable?. PLoS ONE.

[3] Cañete E.J., Sison-Peña C.M., Jimeno C.A. (2014). Clinicopathological, biochemical, and sonographic features of thyroid nodule predictive of malignancy among adult Filipino patients in a tertiary hospital in the Philippines. Endocrinol. Metab..

[4] Carlé A., Krejbjerg A., Laurberg P. (2014). Epidemiology of nodular goitre. Influence of iodine intake. Best Pract. Res. Clin. Endocrinol. Metab..

RETRACTED

[5] Aydin Y., Besir F.H., Erkan M.E., Yazgan O., Gungor A., Onder E., Coşkun H., Aydin L. (2014). Spectrum and prevalence of nodular thyroid diseases detected by ultrasonography in the western black sea region of turkey. Med. Ultrason..

[6] Ajmal S., Rapoport S., Batlle H.R., Mazzaglia P.J. (2015). The natural history of the benign thyroid nodule: What is the appropriate follow-up strategy?. J. Am. Coll. Surg..

[7] Luo J., McManus C., Chen H., Sippel R.S. (2012). Are there predictors of malignancy in patients with multinodular goiter?. J. Surg. Res..

[8] Akushevich I., Kravchenko J., Ukraintseva S., Arbeev K., Yashin A.I. (2013). Time trends of incidence of age-associated diseases in the us elderly population: Medicare-based analysis. Age Ageing.

[9] Li H., Li J. (2015). Thyroid disorders in women. Minerva. Med..

[10] Huan Q., Wang K., Lou F., Zhang L., Huang Q., Han Y., Sun H., Zhu L., Lin P., Song J., Liu F., Wang Q., Hou W. (2014). Epidemiological characteristics of thyroid nodules and risk factors for malignant nodules: a retrospective study from 6,304 surgical cases. Chin. Med. J..

[11] Chuot C.C., Galukande M., Ibingira C., Kisa N., Fualal J.O. (2014). Iodine deficiency among goiter patients in rural South Sudan. BMC Res. Notes.

[12] Biswas A.B., Das D.K., Chakraborty I., Biswas A.K., Sharma P.K., Biswas R. (2014). Goiter prevalence, urinary iodine, and salt iodization level in sub-Himalayan Darjeeling district of West Bengal, India. Indian J. Public Health.

[13] Diez J.J., Iglesias P. (2014). An analysis of the relative risk for goitre in euthyroid patients with type 2 diabetes. Clin. Endocrinol..

[14] Vander J.B., Gaston E.A., Dawber T.R. (1968). The significance of nontoxic thyroid nodules: Final report of a 15-year study of the incidence of thyroid malignancy. Ann. Intern. Med..

[15] Tunbridge W., Evered D., Hall R., Appleton D., Brewis M., Clark F., Evans J.G., Young E., Bird T., Smith P. (1977). The spectrum of thyroid disease in a community: The Wickham survey. Clin. Endocrinol..

[16] Guo H., Sun M., He W., Chen H., Li W., Tang J., Tang W., Lu J., Bi Y., Ning G. (2014). The prevalence of thyroid nodules and its relationship with metabolic parameters in a Chinese community-based population aged over 40 years. Endocrine.

[17] Knudsen N., Laurberg P., Perrild H., Bülow I., Ovesen L., Jørgensen T. (2002). Risk factors for goiter and thyroid nodules. Thyroid.

[18] Aydin L.Y., Aydin Y., Besir F.H., Demirin H., Yildirim H., Önder E., Dumlu T., Celbek G. (2011). Effect of smoking intensity on thyroid volume, thyroid nodularity and thyroid function: The Melen study. Minerva Endocrinol..

[19] Sousa P.A.M., Vaisman M., Carneiro J.R.I., Guimarães L., Freitas H., Pinheiro M.F.C., Liechocki S., Monteiro C.M.M., Teixeira P.F.S. (2013). Prevalence of goiter and thyroid nodular disease in patients with class iii obesity. Arq. Bras. Endocrinol. Metabol..

RETRACTED

[20] Anil C., Akkurt A., Ayturk S., Kut A., Gursoy A. (2013). Impaired glucose metabolism is a risk factor for increased thyroid volume and nodule prevalence in a mild-to-moderate iodine deficient area. Metabolism.

[21] Führer D., Bockisch A., Schmid K.W. (2012). Euthyroid goiter with and without nodules—Diagnosis and treatment. Dtsch. Arztebl. Int..

[22] Kim M.-H., Park Y.R., Lim D.-J., Yoon K.-H., Kang M.-I., Cha B.-Y., Lee K.-W., Son H.-Y. (2010). The relationship between thyroid nodules and uterine fibroids. Endoc. J..

[23] Arduc A., Dogan B.A., Tuna M.M., Tutuncu Y., Isik S., Berker D., Guler S. (2014). Higher body mass index and larger waist circumference may be predictors of thyroid carcinoma in patients with Hürthle-cell lesion/neoplasm fine-needle aspiration diagnosis. Clin. Endocrinol..

[24] Cappelli C., Castellano M., Pirola I., de Martino E., Gandossi E., Delbarba A., Salvi A., Rosei E.A. (2008). Reduced thyroid volume and nodularity in dyslipidaemic patients on statin treatment. Clin. Endocrinol..

[25] Amihăesei I.C., Chelaru L. (2013). Metabolic syndrome a widespread threatening condition; risk factors, diagnostic criteria, therapeutic options, prevention and controversies: An overview. Rev. Med. Chir. Soc. Med. Nat. Lasi.

[26] Zhang J., Jiang R., Li L., Li P., Li X., Wang Z., Li L., Teng W. (2014). Serum thyrotropin is positively correlated with the metabolic syndrome components of obesity and dyslipidemia in Chinese adolescents. Int. J. Endocrinol..

[27] Cheng T.O. (2004). Metabolic syndrome in China. Circulation.

[28] Tamer G., Mert M., Tamer I., Mesci B., Kilic D., Arik S. (2011). Effects of thyroid autoimmunity on abdominal obesity and hyperlipidaemia. Endokrynol. Pol..

[29] Shinkov A., Borissova A.-M., Kovatcheva R., Atanassova I., Vlahov J., Dakovska L. (2014). The prevalence of the metabolic syndrome increases through the quartiles of thyroid stimulating hormone in a population-based sample of euthyroid subjects. Arq. Bras. Endocrinol. Metabol..

[30] Damasceno D.C., Sinzato Y.K., Bueno A., Dallaqua B., Lima P.H., Calderon I.M., Rudge M.V., Campos K.E. (2013). Metabolic profile and genotoxicity in obese rats exposed to cigarette smoke. Obesity.

[31] Rendina D., de Palma D., de Filippo G., de Pascale F., Muscariello R., Ippolito R., Fazio V., Fiengo A., Benvenuto D., Strazzullo P. (2015). Prevalence of simple nodular goiter and hashimoto’s thyroiditis in current, previous, and never smokers in a geographical area with mild iodine deficiency. Horm. Metab. Res..

RETRACTED

[32] Krishnan E. (2014). Interaction of inflammation, hyperuricemia, and the prevalence of hypertension among adults free of metabolic syndrome: Nhanes 2009–2010. J. Am. Heart Assoc..

[33] You L., Liu A., Wuyun G., Wu H., Wang P. (2014). Prevalence of hyperuricemia and the relationship between serum uric acid and metabolic syndrome in the Asian Mongolian area. J. Atheroscler. Thromb..

